This article has been retracted.

# miR-206 Targets MALAT1 to Suppress Cell Progression of Ectopic Endometrial Stromal Cells in Endometriosis

**DOI:** 10.1155/2022/8094385

**Published:** 2022-01-27

**Authors:** Jinggang Li, Xiaofei Guan, Chongyun Xu, Jingyun Jia, Ling Zhang, Hui Han

**Affiliations:** ^1^Department of Gynecology, Affiliated Hospital of Jining Medical University, Jining 272100, China; ^2^Depatment of Obstetrics, Pingdu People's Hospital, Qingdao 266700, China; ^3^Department of Obstetrics, Wulian Country People's Hospital, Rizhao 262300, China; ^4^Department of Obstetrics, Chifeng City Center Hospital Ningcheng Country, Chifeng 024200, China; ^5^Record Room, Gaoqing Country People's Hospital, Zibo 256300, China

## Abstract

**Background:**

miR-206 was reported to be a tumor suppressor in bladder cancer. In this study, we explore the expression and function of miR-206 in endometriosis (EM).

**Methods:**

40 EM patients undergoing total hysterectomy were selected as the experimental group. RT-qPCR assay was adopted to detect the expression of MALAT1 and miR-206 in EM. Cell proliferation was detected by EdU incorporation and colony formation assay. Cell migration and invasion viability of ESCs were examined by transwell assay and wound healing assay. Flow cytometry was carried out to assess cell apoptosis of ESCs. The protein expressions of Bcl-2 and Bax were examined by western blot assay. The relationship between miR-206 and MALAT1 was verified by the dual-luciferase reporter assay and RNA pull-down assay.

**Results:**

In this work, miR-206 was found to be downregulated in EM. Functional experiments displayed that miR-206 mimic repressed cell proliferation, migration, and invasion of ESCs and promoted cell apoptosis of ESCs. Furthermore, miR-206 mimic reduced the expression of Bcl-2 but enhanced the expression of Bax. MALAT1 was found to be upregulated in EM. Furthermore, MALAT1 was indicated to be a target of miR-206. Additionally, MALAT1 was found to alleviate the influence of miR-206 on cell progression of ESCs. Furthermore, miR-206 inhibited tumor growth *in vivo*.

**Conclusion:**

This study indicated that miR-206 inhibited cell progression by regulating MALAT1 in EM. Hence, miR-206 was suggested to be a possible target for EM treatment.

## 1. Introduction

Endometriosis (EM) refers to the infiltration and growth of endometrial tissue outside the uterus [1]. EM is the most common gynecological disease, with progressive aggravation of dysmenorrhea, infertility, and other clinical characteristics of gynecological diseases [2]. EM is hormone-dependent and is more common in women of childbearing age. Although EM is a benign disease, it has behavioral characteristics similar to malignant tumors, such as distant cell metastasis, adhesion, invasion, proliferation, and neovascularization [3]. The origin of ectopic endometrium has not been fully elucidated so far. Therefore, it is urgent to investigate the pathogenesis of EM to search for effective targets.

miRNA, a class of 18–22 nucleotide noncoding single-stranded RNA, controls post-transcriptional gene expression levels by binding to mRNA 3′-UTR [4, 5]. miR-206 was reported to suppress cell migration by downregulating EGFR expression in liver cancer [6]. Additionally, miR-206 promoted mammary differentiation and accumulation of related lipids in breast cancer [7]. Furthermore, miR-206 was at a low level in cervical cancer (CC) and suppressed CC cell invasion, migration, and growth by modulating BAG3 [8]. However, the special effect of miR-206 in EM remains obscure.

lncRNAs are functional RNA molecules over 200 nt in length, lacking the ability to encode proteins and regulating gene expression at various levels [9]. lncRNAs have been increasingly studied in gynecological diseases, including EM. Bai et al. found 1474 differentially expressed lncRNAs in EM by bioinformation technology, and the expressions of RP11-96D and GS1-358P8.4 were closely related to EM cell progression [10]. Furthermore, H19 was found to be a new potential predictor of EM [11]. lncRNA MALAT1 is involved in regulation of gene expression before and after transcription. MALAT1 has been found to be abnormally expressed and plays a key role in a variety of tumors. In ovarian cancer, MALAT1 was found to promote cancer progression by regulating EMT and PI3K/AKT pathway [12]. Furthermore, overexpression of MALAT1 was associated with recurrence of breast cancer [13].

In this study, the expression level of miR-206 was detected in EM. Moreover, the effect of miR-206/MALAT1 on EM progression was also investigated. Overall, miR-206 was suggested to be an effective target for EM treatment.

## 2. Materials and Methods

### 2.1. Clinical Samples

The ectopic endometrial tissues of 40 EM patients undergoing total hysterectomy were selected as the experimental group. In the control group, normal endometrium (NE) tissues were taken from 20 patients excluding those with estrogen-dependent disease during the same period. All tissues were from Affiliated Hospital of Jining Medical University. The average age of patients in the two groups was 37.30 ± 6.83 years and 40.46 ± 5.26 years, respectively. None of the patients had malignant diseases, immune diseases, inflammatory diseases, surgical diseases, and estrogen-dependent diseases. The collection of specimens was informed to the patients and their families and was approved by the Ethics Committee of Affiliated Hospital of Jining Medical University.

### 2.2. Cell Culture and Cell Transfection

The primary endometrial stromal cells (ESCs) were obtained according to previous description. ESCs were cultured in Dulbecco's Modified Eagle Medium (DMEM, Gibco, USA) with 10% fetal bovine serum (FBS, Gibco, USA), 10 U/ml penicillin, and 100U/ml streptomycin at 37°C and 5% CO_2_.

ESCs (1х10^5^ cells/mL) were cultured in a 24-well plate for 24 h. The miR-206 mimic, NC-mimic, miR-206 inhibitor, and NC-inhibitor were obtained from GenePharma (Shanghai, China). pcDNA3.1-MALAT1 and pcDNA3.1-MALAT1 negative control (pcDNA-NC) were obtained from RIBO Bio (Guangzhou, China). Lipofectamine 3000 transfection kit (Invitrogen, USA) was used for cell transfection according to the transfection instructions.

### 2.3. RNA Extraction and RT-qPCR Detection

The total RNAs were obtained by the Trizol Kit (Invitrogen, USA). cDNA was synthesized by PrimeScript RT Reagent Kit gDNA Eraser (Takara, China). RT-PCR assay was performed by using ABI 7500 (Invitrogen, USA). miR-206 expression was measured by MiRx miRNA First Strand Synthesis Kit (TaKaRa Bio, China). The internal reference of miR-206 was U6, and the internal reference of MALAT1 was *β*-actin. All primers (Table 1) were synthesized by Shenggong Biological Engineering (Shanghai, China). The relative expressions of MALAT1 and miR-206 were evaluated by the 2-^△△Ct^ method.

### 2.4. Western Blot Assay

After transfection for 48 h, cells were added with lysate and centrifuged at 10000 r/min for 10 min to obtain total protein. The protein was wet-transferred to PVDF membrane after SDS-PAGE electrophoresis. The membrane was immersed in the primary antibodies at 4°C overnight. Then, the secondary antibodies were incubated for 1 h at room temperature. The primary antibodies were anti-*β*-actin (1 : 1000, #12620, Cell Signaling Technology, MA, USA), anti-Bcl-2 (1 : 1000, #3498, Cell Signaling Technology, MA, USA), anti-Bax (1 : 1000, 14796S, Cell Signaling Technology, MA, USA). The secondary antibodies were anti-rabbit IgG (1 : 2000, #14708, Cell Signaling Technology, MA, USA). Finally, the protein signals were exposed by ECL reagent and gel imaging system.

### 2.5. EdU Incorporation Assay

The cells (2х10^4^/mL) were seeded in 96-well plates in a 37°C incubator. The cells were cultured in serum-free medium for 24 h and then added with EdU. After transfection for 48 h, cell proliferation was examined by EdU assay kit (RiboBio, China).

### 2.6. Colony Formation Assay

Cells were digested with 1% trypsin. After 14 d of culture, the cells were fixed with methanol at room temperature for 15 min and stained with crystal violet at room temperature for 15 min. Olympus Ckx53 inverted phase contrast microscope was adopted to take pictures, and ImageJ (1.48 V) was used to count the number of clones.

### 2.7. Transwell Assay

Cells were seeded in transwell chamber (Corning, USA). After coating the transwell chamber with Matrigel glue (BD Company), cells (2х10^5^/*μ*L) were added to the upper chamber. Then, 600 *μ*L medium with SDF-1 (100 ng/mL) was added to the lower chamber. After cultured at 37°C, 5% CO_2_ for 24 h, the number of cells was counted by the microscope.

### 2.8. Wound Healing Assay

The cells were grown to 90% in a 6-well plate, and then thin scratches were formed by a 10 *μ*L pipette tip. At 0 h and 24 h after scratch, the cell scratch spacing was observed under an optical microscope.

### 2.9. Cell Apoptosis Assay

Cell were resuspended with 1хBinding Buffer. Cells (1х10^6^/mL) were mixed with V-FITC (5 *μ*L) and PI (10 *μ*L). Cell apoptosis rate was detected by flow cytometry after incubation at room temperature for 20 min.

### 2.10. Caspase-3/7 Assay

After transfection, cells were added with Caspase-3/7 regent. After gently shaking the plate for 120 min at room temperature, the luminescence was measured by a plate reading luminometer.

### 2.11. Dual-Luciferase Reporter Assay

TargetScan online software was used to predict the binding sites between miR-206 and MALAT1. Mutant sequences and wild sequence fragments were cloned and combined with Promega vectors. The MALAT1-Mut and MALAT1-Wt were transfected with miR-206 mimic or NC-mimic, respectively. Luciferase activity was detected by dual-luciferase reporter kit.

### 2.12. RNA Pull-Down Assay

Bio-MALAT1-Wt, Bio-MALAT1-Mut, and Bio-NC were obtained from GenePharma (Shanghai, China). After 48 h of transfection with Bio-MALAT1-Wt, Bio-MALAT1-Mut, and Bio-NC, the cells were incubated with Dynabeads M-280 Streptavidin (Invitrogen, USA). RT-qPCR was used to examined the enrichment of miR-206.

### 2.13. Establishment of EM Rat Model

Male rats (BALB/C, 6 weeks old) were raised in SPF level environment. The rat model of EM was established by endometrial transplantation. The rats were divided into 4 groups randomly: the NC-mimic + pcDNA-NC group, miR-206 mimic + pcDNA-NC group, NC-mimic + pcDNA-MALAT1 group, and miR-206 mimic + pcDNA-MALAT1 group, with 6 rats in each group. After injecting the transfected cells, the weight of the rats was assessed weekly. After 4 weeks, the tumors were photographed and weighed.

### 2.14. Statistical Analysis

The data were presented as mean ± SD. SPSS 22.0 and GraphPad Prism 7.0 were used for data analysis. Comparisons between the two groups were assessed by the *t*-test. Additionally, comparisons among multiple groups were compared by one-way ANOVA. It is considered as statistically significant when *P* < 0.05.

## 3. Results

### 3.1. miR-206 Was Downregulated in EM

To explore the effect of miR-206 in EM, miR-206 expression in EM was firstly assessed by RT-qPCR assay. We noticed that miR-206 was remarkably lowly expressed in EM tissues compared with NE tissues (Figure 1(a)). Similarly, miR-206 was at a lower level in ESCs than in NE cells (Figure 1(b)).

### 3.2. miR-206 Inhibited ESC Proliferation in ESCs

To explore the role of miR-206 on cell proliferation in ESCs, miR-mimic or miR-inhibitor was transfected into ESCs (Figure 2(a)). Then, EdU incorporation assay and colony formation assay were used to measure ESC proliferation. Obviously, the results displayed that miR-206 mimic impeded cell proliferation, but miR-206 inhibitor facilitated cell proliferation (Figure 2(b)). Similarly, the number of clones in ESCs was decreased by miR-206 mimic, while it was increased by miR-206 inhibitor (Figure 2(c)). All data indicated that miR-206 mimic repressed ESC growth.

### 3.3. miR-206 Blocked Cell Metastasis in ESCs

Next, the number of migrated cells was clearly declined by miR-206 mimic but accelerated by miR-206 inhibitor (Figure 3(a)). Additionally, miR-206 mimic inhibited scratch healing rate, whereas the contrary effect was exhibited by miR-206 inhibitor (Figure 3(b)). Hence, our results demonstrated that miR-206 blocked ESC metastasis.

### 3.4. miR-206 Facilitated Cell Apoptosis in ESCs

We noticed that miR-206 mimic notably promoted cell apoptosis, but miR-206 inhibitor had an inhibition effect on cell apoptosis (Figure 4(a)). Western blot assay displayed that Bax expression was increased by miR-206 mimic but reduced by miR-206 inhibitor (Figures 4(b) and 4(c)). Inversely, Bcl-2 expression was suppressed by miR-206 mimic, while it was increased by miR-206 inhibitor (Figures 4(b) and 4(c)). Furthermore, miR-206 mimic promoted the Caspase-3/7 activity, whereas miR-206 inhibitor had the opposite effect on Caspase-3/7 activity (Figure 4(d)). Taken together, miR-206 was verified to promote cell apoptosis in ESCs.

### 3.5. miR-206 Negatively Targeted MALAT1

First, MALAT1 was notably higher in EM tissues and ESCs than in NE groups (Figures 5(a) and 5(b)). Furthermore, MALAL1 was negatively correlated with miR-206 expression (Figure 5(c)). TargetScan was used to screen the potential binding sites between MALAT1 and miR-206 (Figure 5(d)). Then, dual-luciferase reporter assay and RT-qPCR assay were adopted to verify this hypothesis. miR-206 mimic suppressed the luciferase activity of MALAT1-Wt, but not MALAT1-Mut (Figure 5(e)). Furthermore, RNA pull-down confirmed that miR-206 directly binds to MALAT1-Wt (Figure 5(f)). Additionally, the expression of MALAT1 was reduced by miR-206 mimic but was increased by miR-206 inhibitor (Figure 5(g)). MALAT1 expression was notably accelerated by pcDNA-MALAT1 (Figure 5(h)). Hence, miR-206 was proved to be a target of MALAT1.

### 3.6. miR-206 Suppressed Cell Progression by Regulating MALAT1 in ESCs

To investigative the function of MALAT1/miR-206 on cell progression in ESCs, pcDNA-MALAT1 was transfected with miR-206 mimic. Cell proliferation was inhibited by miR-206 mimic, while pcDNA-MALAT1 effectively alleviated the inhibition of miR-206 mimic (Figure 6(a)). As we expected, pcDNA-MALAT1 effectively moderated the inhibition of miR-206 mimic on cell clones (Figure 6(b)). Similarly, cell migration and invasion ability were inhibited by miR-206 mimic, whereas the inhibition of miR-206 mimic on cell migration and invasion was impaired by pcDNA-MALAT1 (Figures 6(c) and 6(d)). Therefore, miR-206 suppressed cell progression by regulating MALAT1 in ESCs.

### 3.7. miR-206 Hampered Tumor Growth by Regulating MALAT1 In Vivo

To explore the function of miR-206 on EM progression in vivo, ESCs transfected with paDNA-MALAT1and miR-206 mimic were injected into the rat EM model. We took out the tumor every one week for photographing and weighing. The results revealed that pcDNA-MALAT1promoted tumor growth, while miR-206 mimic inhibited the effect of pcDNA-MALAT1 on tumor growth (Figures 7(a), 7(c), and 7(d)). After 4 weeks, the tumor weight was significantly increased by pcDNA-MALAT1, whereas miR-206 mimic weakened the effect of pcDNA-MALAT1 (Figure 7(b)). Hence, all data indicated that miR-206 restrained tumor growth by regulating MALAT1 expression in vivo.

## 4. Discussion

Increasing evidences have displayed that miRNAs play a vital role in the pathological development of EM. For instance, miR-202-3p repressed EM cell growth and invasion and induced cell apoptosis by regulating YAP1 [14]. Zhao et al. found that miR-194-5p repressed cell progression and promoted cell apoptosis of ectopic endometrial cells by modulating STAT1/mTOR signaling pathway [15]. Moreover, exosomal miR-214-3p suppressed cell fibrosis in EM by targeting CCN2, suggesting that miR-214-3p may be a biomarker for EM therapy [16]. miR-206 has been reported to be a therapy biomarker in CC [17]. In the current work, miR-206 was found to be downregulated in EM and ESCs. In line with our findings, the expression of miR-206 showed a downward trend in hepatocellular carcinoma [18], head and neck squamous cell carcinoma [19], and lung cancer [20]. Next, functional experiments indicated that forced expression of miR-206 restrained cell proliferation, migration, and invasion of ESCs. Besides that, miR-206 mimic enhanced cell apoptosis of ESCs. Previous studies have reported that miR-206 was a tumor-inhibiting factor in CC [8]. Similar to our results, miR-206 blocked cell proliferation, lactate production, and glucose consumption in colon cancer [21]. Furthermore, miR-206 was found to restrict cell proliferation and metastasis by negatively regulating CORO1C in non-small-cell lung cancer [22].

Numerous studies have found that lncRNAs play a vital role in EM by targeting miRNAs. Knockdown of lncRNA AFAP1-AS1 blocked ESC growth by targeting miR-424-5p [23]. LINC01541 suppressed cell progression of ESCs, but miR-506-5p impaired its inhibiting effect [24]. MALAT1 was found to accelerate the cell processes in EM by targeting miR-200c [25]. In our study, we found that miR-206 interacted with MALAT1. Moreover, MALAT1 was upregulated in EM and ESCs and alleviated the effect of miR-206 on ESC progression. Sun et al. reported that MALAT1 facilitated cell differentiation by sponging miR-206 in bone marrow-derived mesenchymal stem cells [26]. Moreover, MALAT1 facilitated cell progression by targeting miR-206 and regulating CDK9 in osteosarcoma [27]. MALAT1 silencing suppressed cell progression by targeting miR-206/VEGFA in hemangioma endothelial cells [28]. Additionally, miR-206 was demonstrated to suppress tumor growth by regulating MALAT1 expression in vivo.

## 5. Conclusion

Our data indicated that miR-206 overexpression repressed cell progression and promoted cell apoptosis by targeting MALAT1. We suggest that miR-206 might be an effective biomarker for EM therapy.

## Figures and Tables

**Figure 1:** miR-206 was downregulated in EM. (a) The expression of miR-206 was downregulated in EM and NE tissues. (b) The expression of miR-206 was lower in ESCs than in NE cells. ^*∗*^*p* < 0.05; ^*∗∗*^*p* < 0.01.

**Figure 2:** miR-206 inhibited cell proliferation in ESCs. (a)The expression of miR-206 was significantly increased by miR-206 mimic, while it was reduced by miR-206 inhibitor. (b) Cell proliferation was suppressed by miR-206 mimic, while it was promoted by miR-206 inhibitor. (c) miR-206 mimic reduced the number of colonies, whereas miR-206 inhibitor increased the number of colonies. ^*∗*^*p* < 0.05; ^*∗∗*^*p* < 0.01.

**Figure 3:** miR-206 inhibited cell migration and invasion in ESCs. (a) Cell migration was inhibited by miR-206 mimic, but it was promoted by miR-206 inhibitor (magnification, 200×). (b) Cell invasion was suppressed by miR-206 mimic, while it was facilitated by miR-206 inhibitor. ^*∗*^*p* < 0.05; ^*∗∗*^*p* < 0.01.

**Figure 4:** miR-206 promoted cell apoptosis in ESCs. (a) miR-206 mimic promoted cell apoptosis, while miR-260 inhibitor suppressed cell apoptosis. (b, c) The protein expressions of Bax and Bcl-2 were detected by western blot assay. (d) miR-206 mimic increased Caspase-3/7 activity, while miR-206 inhibitor declined Caspase-3/7 activity. ^*∗*^*p* < 0.05; ^*∗∗*^*p* < 0.01.

**Figure 5:** MALAT1 acted as a target of MiR-206. (a) MALAT1 was significantly upregulated in EM. (b) The expression of MALAT1 was high in ESCs. (c) There was a negative correlation between miR-206 and MALAT1. (d) There were special binding sites between miR-206 and MALAT1. (e) miR-206 mimic reduced the luciferase activity of MALAT1-Wt but had no effect on MALAT1-Mut. (f) The combining capacity between miR-206 and MALAT1 was detected by RNA pull-down. (g) MALAT1 expression was inhibited by miR-206, while it was promoted by miR-206 inhibitor. (h) MALAT1 expression was significantly increased by pcDNA-MALAT1. ^*∗∗*^*p* < 0.01; ^*∗∗∗*^*p* < 0.001.

**Figure 6:** miR-206 suppressed cell progression by regulating MALAT1 in ESCs. (a) pcDNA-MALAT1 effectively alleviated the inhibition effect of miR-206 mimic on ESC proliferation. (b) pcDNA-MALAT1 effectively alleviated the inhibition of miR-206 mimic on ESC cloning. (c, d) pcDNA-MALAT1 effectively alleviated the inhibition of miR-206 mimic on ESC migration and invasion (magnification, 200×). (e) pcDNA-MALAT1 effectively inhibited the apoptosis of ESCs after transfection with miR-206 mimic. (f) Western blot assay was used to detect the protein expression levels of apoptosis-related proteins (Bcl-2 and Bax). (g) Caspase-3/7 activity was detected in ESCs transfected with pcDNA-MALAT1 or miR-206. ^*∗*^*p* < 0.05; ^*∗∗*^*p* < 0.01; ^#^*p* < 0.05 vs. miR-206 mimic + pcDNA-NC group or NC-mimic + pcDNA-MALAT1 group.

**Figure 7:** miR-206 inhibited tumor growth by regulating MALAT1 in vivo. (a) Image of ectopic endometrial cysts removed weekly after resection. (b) Weight of ectopic endometrial cyst excised after 4 weeks. (c) Weekly volume of ectopic endometrial cysts. (d) Weekly weight of EM rats. ^*∗*^*p* < 0.05; ^*∗∗*^*p* < 0.01; ^*∗∗∗*^*p* < 0.001; ^#^*p* < 0.05; ^###^*p* < 0.001 vs. NC-mimic + pcDNA-MALAT1 group or miR-206 mimic + pcDNA-NC group.

**Table 1:** Primer sequences in RT-qPCR.

Gene		Sequences 5′-3′
miR-206	Forward	5′- CAGATCCGATTGGAATGTAAGG-3′
	Reverse	5′- TATGClTGlTrCTCGTCTCTGTGTC-3′
MALAT1	Forward	5′- AAAGCAAGGTCTCCCCACAAG-3′
	Reverse	5′- GGTCTGTGCTAGATC-3′
U6	Forward	5′- ATTGGAACGATACAGAGAAGATT-3′
	Reverse	5′- GGAACGCTTCACGAATTTG-3′
*β*-Actin	Forward	5′- GGTGGTCTCCTCTGACTTCAACA-3′
	Reverse	5′- CTTGCTGTAGCCAAATFCGTTGT-3′

## Data Availability

The data used to support the findings of this study are available on reasonable request from the corresponding author.
